The article "Cognitive IoT-Based e-Learning System: Enabling Context-Aware Remote Schooling during the Pandemic" was retracted in 2023. Reasons: signs of a paper mill; suspected computer-generated content; unreliable results or conclusions; concerns about the data.

# Cognitive IoT-Based e-Learning System: Enabling Context-Aware Remote Schooling during the Pandemic

**DOI:** 10.1155/2021/7358874

**Published:** 2021-08-31

**Authors:** Atef Zaguia, Darine Ameyed, MohamedAmime Haddar, Omar Cheikhrouhou, Habib Hamam

**Affiliations:** ^1^Computer Sciences Department, College of CIT, Taif University, P.O. Box 11099, Taif 21944, Saudi Arabia; ^2^System Engineering Department, Ecole de Technologie Supérieure, University of Quebec, Montreal, Canada; ^3^Information Technology Department, College of CIT, Taif University, P.O. Box 11099, Taif 21944, Saudi Arabia; ^4^Faculty of Engineering, Uni de Moncton, New Brunswick, Canada; ^5^School of Elect. Eng. and Electronic Eng., University of Johannesburg, Johannesburg, South Africa; ^6^CES Laboratory National School of Engineers of Sfax, University of Sfax, Sfax 3038, Tunisia

## Abstract

The 2019–2020 coronavirus pandemic had far-reaching consequences beyond the spread of the disease and efforts to cure it. Today, it is obvious that the pandemic devastated key sectors ranging from health to economy, culture, and education. As far as education is concerned, one direct result of the spread of the pandemic was the resort to suspending traditional in-person classroom courses and relying on remote learning and homeschooling instead, by exploiting e-learning technologies, but many challenges are faced by these technologies. Most of these challenges are centered around the efficiency of these delivery methods, interactivity, and knowledge testing. These issues raise the need to develop an advanced smart educational system that assists home-schooled students, provides teachers with a range of smart new tools, and enable a dynamic and interactive e-learning experience. Technologies like the Internet of things (IoT) and artificial intelligence (AI), including cognitive models and context-awareness, can be a driving force in the future of e-learning, opening many opportunities to overcome the limitation of the existing remote learning systems and provide an efficient reliable augmented learning experience. Furthermore, virtual reality (VR) and augmented reality (AR), introduced in education as a way for asynchronous learning, can be a second driving force of future synchronous learning. The teacher and students can see each other in a virtual class even if they are geographically spread in a city, a country, or the globe. The main goal of this work is to design and provide a model supporting intelligent teaching assisting and engaging e-learning activity. This paper presents a new model, ViRICTA, an intelligent system, proposing an end-to-end solution with a stack technology integrating the Internet of things and artificial intelligence. The designed system aims to enable a valuable learning experience, providing an efficient, interactive, and proactive context-aware learning smart services.

## 1. Introduction

The Internet has created a globalized world in which people consume, produce, and communicate information in different ways overcoming physical boundaries limitations. Broadband connectivity access and rapid technological development led to exponential adoption of digital solutions in many sectors. The beginning of the 21st century witnessed the emergence of e-learning platforms. This encouraged education leaders to push learning beyond school walls and engage people in lifelong learning journeys. For instance, e-learning comes as a solution for most of the learning constraints such as lack of time and resources.

e-Learning is an integrated system based on the effective employment of Information and Communication Technology (ICTs) in the teaching and learning processes by creating an environment rich in computer and Internet applications that enables the learner to access the learning resources anytime and anywhere and to achieve mutual interaction between the elements of the system [1]. e-Learning is the most commonly used term. We also use other terms such as electronic education or online learning or virtual learning. e-Learning [2] is based on electronic education systems such as computer education systems, video-conference systems, and the related concepts including virtual reality, interactive video, and e-books. The literature divides e-learning into three crucial types:

- Synchronous e-learning: this is a kind of education that requires both learners and teachers to have direct interaction, such as exchanging ideas between them through chatting or virtual classes
- Asynchronous e-learning: this type does not require the teacher and learner to meet; the learner can interact with the educational content and interact through traditional methods such as e-mail or through the use of specialized software based on the multiple multimedia system
- Built-in education: education depends on the combination of simultaneous and asynchronous e-learning

Over the last decade, e-learning has shown significant growth, as the Internet, technologies, and education combine to provide people with the opportunity to gain new skills. Since the COVID-19 outbreak, most governments around the world have closed educational institutions in an attempt to contain the spread of the virus. Globally, over 1.2 billion children are out of the classroom. This underlines why online learning has become more important in people's lives. As a result, education has changed dramatically, with the distinctive rise of e-learning, whereby teaching is undertaken remotely and on digital platforms. Even before the pandemic, there was already high growth and adoption in education technology with global investment reaching 18.66 billion US dollars and markets forecast the online education as 350 billion dollars industry by 2025, which might be updated after analyzing the impacts of COVID-19 [3] on the online learning market.

Online learning is becoming a huge catalyzer for people and companies to help the adoption of the dynamic and fast change in the world. As they provide many advantages such as time convenience or being cost-friendly, the online courses offer a more affordable option than traditional systems. Despite the rapid adoption and development of e-learning, the e-learning system, platforms, and solutions still face many issues to improve the users-centered experiences.

Context-awareness enhances the system's capabilities to enable the learning environment by intelligent monitoring and adaptability to the user's needs with awareness to his environment based on real-world observation considering the user's specific context. Furthermore, including intelligent modules and supporting different human-machine interaction approaches based on IoT [4, 5] and ambient intelligence can help provide an efficient learning experience. Thus, we aim to enhance the e-learning systems with context-awareness capabilities and intelligent modules to assist its users.

In this paper, we propose an IoT-based smart learning system architecture, including entity-based model and its function view incorporating the context-awareness modules. We also present the model's implementation plan supported by a simulation to prove the concept and functionality of the proposed system.

The paper is structured as follows: in the Related Work section, we overview the state of the art in the e-learning existing systems. Then, we introduce our approach by presenting the architecture's entity-based model and its functional view. Thereafter, we explain the deployment and we prove the concept of our model. Next, we validate through a simulation, we present and discuss the results, and we finish by a conclusion and future works.

## 2. Related Work

During the last decade, the domain of e-learning has grown quite fast. Many known learning management systems (LMSs) were implemented and diversified enjoying the reliance on various methodologies and efficient algorithmic developments [6–8]. In such systems, an e-learning environment will be shared to the learners through their personal devices. These systems enable learners to interact and collaborate with other learners and teachers to realize their assessments and a specific educational task. These systems are characterized by the ability to interact in the harmonious way with the learners [9].

The authors in [10] presented an online system used at the International University of La Rioja that has about 30,000 enrolled students. The online system is a remote virtual laboratory, which provides a practical education by using tools for experimentation in engineering education. The instructor can move from one online working space to another to help students solve their lab instructions. This system is essentially used to offer online laboratories. However, this system does not take into consideration the interaction and the student's contexts.

The authors of [11–14] presented e-learning systems enabling the users to chat, talk, and share information including video, shared applications, and audio. These systems are not conceived to be smart and user-centered. The authors of [1, 2, 15–18] proposed the use of the context-awareness system collecting a large volume of information about the learner's environment. According to these data, the system will automatically adapt to the user's preferences. The integration of the context-awareness in the e-learning system will be an efficient technique to enhance learning.

The authors in [19–24] suggested using artificial intelligence (AI) techniques, such as data mining and fuzzy logic, to enhance the e-learning strategies with a smart way and augment interactions between learners. Most of these systems limit the context to the learner's assessment score, the time needed to complete the assessment test, histories, etc.

The study in [14] highlighted the use of smart mobile devices (SMD) in e-learning. Distance learning platforms (DLP) must integrate these devices. These devices became more and more accessible to the public and easier to use. The authors propose a three-layer platform which consists of an intelligent agent installed on the student smart device. This layer collects all the necessary information related to the student behavior, preoccupations, involvement in the course, etc. and sends it to the second layer. The second layer analyzes the student information, feedback, and rating of course materials using AI techniques and proposes adequate course content. This work proposes the use of smart devices assessing the learner behavior to provide adequate course material personalization.

As explained earlier in related works, with the growth of technological expansion, the e-learning solution is incessantly improving in terms of effectiveness and efficiency. It is also gaining ground, especially during the COVID-19 crisis, and it is expected to be widely used in the post-COVID-19 era. However, the existing solution still faces many challenges to be more learner-centered. They do not automatically and dynamically adapt to the user's context and his changing environment to provide adequate services. For instance, on the one hand, these systems did not prove to be efficient to reveal the students' identity and check their attendance during a remote course or exam. On the other hand, they did not ensure that the student was getting academic achievement.

The existing e-learning platforms and systems still face a lack of multiple key factors for a successful, efficient, and customized learning experience. We mention as an example the lack of (i) an immersive experience, (ii) smart assistance for the learning activity, (iii) efficient interactivity between the students and the learning provider, and (iv) services proactivity including predicting the needs of the users. These limits should be overcome while ensuring a transition from e-learning to smart learning. This transition can be enabled by context-awareness, an IoT-based monitoring approach, and intelligent modules for users' assistance. In the present work, we propose an architecture framework supporting a smart e-learning environment. Our main goal is to enhance the learning experience by a user-centered system, in which we incorporate a deep awareness of the physical and logical user's context. The following section will explain and describe our proposed model.

## 3. The Planned Proposed System: ViRICTA

Students' interaction and collaboration over the learning process are crucial for an efficient experience. Using the Internet of things (IoT) can help enhance the interactivity and understand the student context. Also, determining student concentration is an essential part of educational assessment, as the student behaviors are indicative of the student's cognitive activity, and this behavior can be used as a measurement of engagement recognition. In our framework, we propose to incorporate a sensing layer into the e-learning platform to gather physical, ambient, and behavioral data. These data help extend the platform to a pervasive learning system including context-awareness capacities. We also embedded cognitive modules to extract valuable knowledge to conduct smart services aligned with the user's needs. We start by presenting the IoT-entity view which presents the architecture's models components and its relations. Then, we present the function view to explain the different running process and functionalities supported by the proposed models.

### 3.1. Architecture Model IoT-Based Smart Learning

In this section, we will illustrate the architectural framework of our proposed system model IoT-based smart learning. First, we will describe our IoT-entity model-based smart learning and then the IoT smart learning system deployment view.

#### 3.1.1. IoT-Entity Model-Based Smart Learning

As shown in the diagram (Figure 1), the IoT entity-based smart learning consists of the following elements (starting from the entities at the bottom):

(1) Physical entities (student environment professor environment) are the real-world things that are operated and sensed upon by the IoT devices.
(2) Student environment professor environment represents different types of materials that can be attached to the workstations of both the student and professor to aid in their monitoring and identification.
(3) IoT devices, for both the student and professor, interact with the physical world via sensing and actuation. They communicate through a network. IoT devices include the following:
  - Sensors, observe a property of a physical entity, in our case the workstation, and convert it to human readable form: digital information. For instance, the IoT sound sensor will detect the noise level and according to this information, the system will interact.
  - Actuators act on or change some properties of the physical entities based on digital instructions.
(4) The module IoT gateway unfolds two main modules: the *edge* module and the *networking* module. The *edge* module supports local processing capability. It operates on data coming from the IoT devices and operates according to that information. The *networking* module deals with communication.
(5) The operation and management subsystem: those modules provide access point to the system managers to help maintain the overall good operation of the IoT systems. It incorporates the main functions responsible for provisioning, managing, monitoring, and optimizing the general systems' operational performance. It includes operation support system and application support system.
(6) Resource access interchange subsystem: it encloses the controlled end-points offering services to the users of the IoT system interacting via their devices and peer system. It helps gate them to the IoT system's capabilities.
(7) Application service subsystem: this module will include all the adequate services that can be afforded to the user in the context of smart learning. More details will be presented in the services section.
(8) IoT-users (students and professor) interact with the smart learning system using devices, such as personal computers, tablets, smartphones, or a more specialized device. To help or assist the user in an effective way, these devices will be equipped with a special user interface to facilitate the smart learning.

### 3.2. Services Function View

As shown in Figure 2, the IoT smart learning system services consist of the following elements.

#### 3.2.1. Course Material

This module will contain the course materials. It will be updated by the teacher. It will provide the adequate materials to the students.

#### 3.2.2. Face Recognition and Emotion Face-Based Recognition

The goal of this module is to detect the identity, the presence, and the status of the user. For instance, this module will detect if the student, during revision, is focused on 1 slide too long. In this case, he has a problem understanding this slide; therefore, an alert will be sent to the student to determine if he needs exercises or more help.

#### 3.2.3. Help History Community

The aim of this module is to provide help to the student, if needed, through the students community.

#### 3.2.4. Student Portfolio

This module will record the preference, the history, and the weak and the strong points of the student, to take it into consideration to improve the level of the student.

#### 3.2.5. Context-Awareness

The aim of this module is to provide adequate services to the student according to the context. Context-awareness is a main concept in pervasive and ubiquitous computing. In context-aware systems, information can be collected by using tiny resource-bounded devices, such as PDAs, smart phones, wireless sensors, and connected objects. This allows a better understanding of the service context and the user needs which help provide an efficient assistance on the user activity.

#### 3.2.6. Assessment and Evaluation

This module sends notifications to the students to notify them about the date of the exams and assessments.

## 4. Deployment Plan, Proof of Concept, and Results

### 4.1. IoT Smart Learning System Deployment View

The depiction of the IoT smart learning system deployment view (Figure 3) is as follows.

#### 4.1.1. Physical Entity Domain

This mainly consists of sensed physical objects and controlled physical objects, which are related to IoT applications and are of interest to users. A sensed physical object is a physical entity, from which information is acquired by sensors, while a controlled physical object is a physical entity which is subject to actions of actuators. In our system, we have 2 different workstations: student environment and professor environment.

#### 4.1.2. Sensing Controlling Domain

It is essentially composed of three entities: actuators, sensors, and IoT gateway. Depending on the information collected by the sensors, the IoT gateway will take the adequate decision and send the actions to actuators.

Application service domain: this domain includes all the adequate services that can be afforded to the user in the context of smart learning. More details will be presented in the services section.

#### 4.1.3. Operation and Management Domain

It includes device registry data store and associated devices identity services and devices management application providing access control, administration, and business capabilities.

#### 4.1.4. Resource Access Interchange Domain

This domain supports access capabilities for users and peers' systems.

#### 4.1.5. User Domain

The user domain contains both student/professor users and digital users. Digital users are devices of some type and they interact directly with other entities in the IoT system via user interfaces. Student/professor users interact using a user device which contains some form of HCI.

### 4.2. Simulation

In our smart learning system, the steps of each strategy are evaluated by developing a simulation model as presented in Figure 4. To simulate our model, we used CPN Tools. CPN Tools is an advanced tool for editing, simulating, and analyzing colored Petri nets. The diagram in Figure 4 illustrates the intricate Petri net demonstrating various states and transitions. Our model is designed depending on the architecture presented in Figure 1.

Normally, a class is based upon teacher-students interactions. The course is performed via slides. Every set of slides presents a subject or LLOs (learning lecture outcomes). In our case, the online class stipulates a professor and 16 students interacting for 1 hour. The class will deal with 6 subjects or 6 LLOs (learning lecture outcomes) taking approximately 10 minutes each. During the performance of each subject, the system will randomly generate the state of the student and his environment.

For every student, the simulation will go initially by the transition “physical entity student,” then “IoT devices,” after the transition “IoT gateway,” and finally the transition “application service subsystem” which will transmit the adequate decisions to the student and the professor.

The aim of the transaction physical entity student is to randomly generate the learning context of the student. As shown in Figure 5, usually the learning contexts are assignment, course, revision, or none. In our case, to simulate our model, we limited it to the “course” context learning.

The transition “IoT device” will generate for every student his states and his environmental contexts. As shown in Figure 6, the system will randomly generate the noise level, temperature level, and luminosity level for the environmental context and it will generate the user context, user state, and user stress. Tables 1 and 2 illustrate the different contexts generated by the system during every subject. This information will be sent to “IoT gateway” transition.

### 4.3. Results and Discussion

Table 3 presents a part of the local decision taken by the transition “IoT gateway” concerning student 5. It summarizes the different notifications sent to student 5 according to the information collected in Tables 1 and 2. For instance, as shown in Table 1, during the presentation of subject 1 the level of the luminosity is too low; (1) therefore the message “turn on light” was sent to student 5; also, during the presentation of subject 5, the level of the noise is too high (8) and the level of the luminosity is low (2) so the messages “decrease noise” and “turn on light” were sent to the student. Additionally, during the presentation of subject 6, the system detects that the student is stressed, so a message to relax was sent to the student.

Figure 7 summarizes the rate of students who fully grasped each of the subjects. These rates were calculated by the transition “application service subsystem” from the information gathered from “IoT gateway” (Tables 1 and 2).

As shown in Figure 7, for instance, 43.75% of the students have grasped subject 1. This rate is too low; therefore, the professor needs to take adequate decisions.

The information presented in Figure 7 permits the professor to get details about every lecture and the rate of the students understanding to make improvement for the next lecture and prepare more exercises for these students.

To conclude, our system will be a remarkable leap towards the cutting edge of the efficiency of online learning. It will make it feasible for the professor to watch his learners' progress, weaknesses, attendance, etc. and, therefore, assign remedial tasks and activities.

## 5. Conclusions

The 2019–2020 coronavirus pandemic uncovered the problems of existing e-learning systems. Learning capabilities and concentration of young students who used to learn in physical school have notably decreased. The major problem of existing systems is the inability of the teacher to control the students' behavior during the lectures. Young students acquire more freedom to behave while the teacher is explaining the lessons. Thus, this results in a lot of misunderstanding leading to a notable degradation of the students' marks.

In this paper, we proposed a new smart e-learning framework that focuses on synchronous e-learning for students. This framework proposes a new way of distant learning, in which the teacher acquires a larger control on learners. IoT, AI, and VR tools are combined together to build a stronger system that helps the teacher supervise the students while presenting lessons and during exams. Future extensions of our systems are mainly related to more computer-aided services to help the teacher discover and react to the students' behavior.

## Figures and Tables

**Figure 1:** Entity-based IoT smart learning.

**Figure 2:** IoT smart learning system services.

**Figure 3:** IoT smart learning system deployment view.

**Figure 4:** Framework of the smart learning system with CPN.

**Figure 5:** Context learning generator.

**Figure 6:** IoT-based sensing and controlling context.

**Figure 7:** The rate of students who fully grasped each of the subjects.

**Table 1:** Different contexts generated: subjects 1, 2, and 3.

	Subject 1	Subject 2	Subject 3
Student 1	Noise level: **6**	Noise level: **3**	Noise level: **9**
	Luminosity level: **2**	Luminosity level: **7**	Luminosity level: **3**
	State: **understanding**	State: **understanding**	State: **not present**
	Stress: **normal**	Stress: **normal**	Stress: **stress**

Student 2	Noise level: **2**	Noise level: **6**	Noise level: **3**
	Luminosity level: **4**	Luminosity level: **2**	Luminosity level: **5**
	State: **not concentrating**	State: **understanding**	State: **understanding**
	Stress: **normal**	Stress: **normal**	Stress: **stress**

Student 3	Noise level: **8**	Noise level: 7	Noise level: **7**
	Luminosity level: **3**	Luminosity level: **8**	Luminosity level: **10**
	State: **not present**	State: **not present**	State: **not concentrating**
	Stress: **stress**	Stress: **normal**	Stress: **normal**

Student 4	Noise level: **5**	Noise level: **2**	Noise level: **6**
	Luminosity level: **9**	Luminosity level: **9**	Luminosity level: **2**
	State: **not understanding**	State: **not concentrating**	State: **not present**
	Stress: **normal**	Stress: **normal**	Stress: **normal**

Student 5	Noise level: **6**	Noise level: **6**	Noise level: **4**
	Luminosity level: **1**	Luminosity level: **10**	Luminosity level: 1**0**
	State: **understanding**	State: **not present**	State: **not concentrating**
	Stress: **normal**	Stress: **normal**	Stress: **stress**

Student 6	Noise level: **1**	Noise level: **2**	Noise level: **5**
	Luminosity level: **7**	Luminosity level: **4**	Luminosity level: **1**
	State: **understanding**	State: **not present**	State: **understanding**
	Stress: **stress**	Stress: **stress**	Stress: **normal**

Student 7	Noise level: **4**	Noise level: **8**	Noise level: **3**
	Luminosity level: **2**	Luminosity level: **5**	Luminosity level: **3**
	State: **not present**	State: **understanding**	State: **not present**
	Stress: **stress**	Stress: **stress**	Stress: **stress**

Student 8	Noise level: **7**	Noise level: **9**	Noise level: **2**
	Luminosity level: **5**	Luminosity level: **8**	Luminosity level: **7**
	State: **not present**	State: **understanding**	State: **understanding**
	Stress: **stress**	Stress: **normal**	Stress: **normal**

Student 9	Noise level: **9**	Noise level: **6**	Noise level: **10**
	Luminosity level: **2**	Luminosity level: **6**	Luminosity level: **4**
	State: **understanding**	State: **not understanding**	State: **understanding**
	Stress: **normal**	Stress: **stress**	Stress: **normal**

Student 10	Noise level: **1**	Noise level: **8**	Noise level: **2**
	Luminosity level: **5**	Luminosity level: **5**	Luminosity level: **10**
	State: **not concentrating**	State: **not present**	State: **not concentrating**
	Stress: **stress**	Stress: **stress**	Stress: **stress**

Student 11	Noise level: **4**	Noise level: **2**	Noise level: **3**
	Luminosity level: **1**	Luminosity level: **10**	Luminosity level: **6**
	State: **not understanding**	State: **not concentrating**	State: **understanding**
	Stress: **stress**	Stress: **normal**	Stress: **stress**

Student 12	Noise level: **5**	Noise level: **6**	Noise level: **8**
	Luminosity level: **3**	Luminosity level: **1**	Luminosity level: **4**
	State: **understanding**	State: **understanding**	State: **not present**
	Stress: **normal**	Stress: **normal**	Stress: **normal**

Student 13	Noise level: **3**	Noise level: **9**	Noise level: **6**
	Luminosity level: **6**	Luminosity level: **7**	Luminosity level: **10**
	State: **not concentrating**	State: **not understanding**	State: **understanding**
	Stress: **stress**	Stress: **stress**	Stress: **stress**

Student 14	Noise level: **3**	Noise level: **1**	Noise level: **8**
	Luminosity level:	Luminosity level: **3**	Luminosity level: **1**
	State: **understanding**	State: **understanding**	State: **understanding**
	Stress: **normal**	Stress: **stress**	Stress: **normal**

Student 15	Noise level: **3**	Noise level: **2**	Noise level: **9**
	Luminosity level: **1**	Luminosity Level:**10**	Luminosity level: **5**
	State: **understanding**	State: **not understanding**	State: **not concentrating**
	Stress: **normal**	Stress: **stress**	Stress: **stress**

Student 16	Noise level: **4**	Noise level: **1**	Noise level: **3**
	Luminosity level: **4**	Luminosity level: **3**	Luminosity level: **5**
	State: **not understanding**	State: **not understanding**	State: **not present**
	Stress: **stress**	Stress: **normal**	Stress: **normal**

Bold indicates the values of the different context parameters detected randomly by IoT devices.

**Table 2:** Different contexts generated: subjects 4, 5, and 6.

	Subject 4	Subject 5	Subject 6
Student 1	Noise level: 3	Noise level: **8**	Noise level: **5**
	Luminosity level: 10	Luminosity level: **4**	Luminosity level: **7**
	State: **understanding**	State: **not present**	State: **not concentrating**
	Stress: **normal**	Stress: **normal**	Stress: **stress**

Student 2	Noise level: **5**	Noise level: **6**	Noise level: **8**
	Luminosity level: **8**	Luminosity level: **9**	Luminosity level: **9**
	State: **understanding**	State: **understanding**	State: **not understanding**
	Stress: **normal**	Stress: **stress**	Stress: **normal**

Student 3	Noise level: 1	Noise level: 9	Noise level: **7**
	Luminosity level: 9	Luminosity level: **6**	Luminosity level: **3**
	State: **not concentrating**	State: **understanding**	State: **not concentrating**
	Stress: **stress**	Stress: **normal**	Stress: **stress**

Student 4	Noise level: **8**	Noise level: **5**	Noise level: **6**
	Luminosity level: **7**	Luminosity level: **10**	Luminosity level: **2**
	State: **not present**	State: **not concentrating**	State: **not present**
	Stress: **stress**	Stress: **stress**	Stress: **normal**

Student 5	Noise level: **8**	Noise level: **8**	Noise level: **3**
	Luminosity level: **9**	Luminosity level: **2**	Luminosity level: 9
	State: **understanding**	State: **understanding**	State: **not understanding**
	Stress: **normal**	Stress: **normal**	Stress: **stress**

Student 6	Noise level: **3**	Noise level: **2**	Noise level: **2**
	Luminosity level: **10**	Luminosity level: **4**	Luminosity level: **8**
	State: **understanding**	State: **not understanding**	State: **understanding**
	Stress: **stress**	Stress: **stress**	Stress: **stress**

Student 7	Noise level: **7**	Noise level: **7**	Noise level: **9**
	Luminosity level: **4**	Luminosity level: **3**	Luminosity level: **7**
	State: **understanding**	State: **understanding**	State: **not concentrating**
	Stress: **normal**	Stress: **stress**	Stress: **normal**

Student 8	Noise level: **6**	Noise level: **2**	Noise level: **7**
	Luminosity level: **3**	Luminosity level: **5**	Luminosity level: **4**
	State: **not understanding**	State: **not concentrating**	State: **understanding**
	Stress: **normal**	Stress: **normal**	Stress: **stress**

Student 9	Noise level: **7**	Noise level: **9**	Noise level: **1**
	Luminosity level: **10**	Luminosity level: **3**	Luminosity level: **3**
	State: **understanding**	State: **not concentrating**	State: **understanding**
	Stress: **stress**	Stress: **stress**	Stress: **stress**

Student 10	Noise level: **3**	Noise level: **8**	Noise level: **2**
	Luminosity level: **2**	Luminosity level: **5**	Luminosity level: **3**
	State: **not present**	State: **not present**	State: **not concentrating**
	Stress: **stress**	Stress: **stress**	Stress: **normal**

Student 11	Noise level: **10**	Noise level: **2**	Noise level: **3**
	Luminosity level: **2**	Luminosity level: **10**	Luminosity level: **6**
	State: **understanding**	State: **not understanding**	State: **not concentrating**
	Stress: **normal**	Stress: **stress**	Stress: **stress**

Student 12	Noise level: **8**	Noise level: **10**	Noise level: **5**
	Luminosity level: **8**	Luminosity level: **8**	Luminosity level: **10**
	State: **not present**	State: **not present**	State: **understanding**
	Stress: **stress**	Stress: **normal**	Stress: **stress**

Student 13	Noise level: **5**	Noise level: **9**	Noise level: **8**
	Luminosity level: **3**	Luminosity level: **7**	Luminosity level: **8**
	State: **understanding**	State: **not present**	State: **understanding**
	Stress: **stress**	Stress: **stress**	Stress: **normal**

Student 14	Noise level: **1**	Noise Level:**10**	Noise level: **7**
	Luminosity level: 9	Luminosity level: **7**	Luminosity level: **3**
	State: **not concentrating**	State: **understanding**	State: **not present**
	Stress: **stress**	Stress: **normal**	Stress: **normal**

Student 15	Noise level: **6**	Noise level: **4**	Noise level: **3**
	Luminosity level: **5**	Luminosity Level:**8**	Luminosity level: **8**
	State: **not understanding**	State: **understanding**	State: **not concentrating**
	Stress: **normal**	Stress: **stress**	Stress: **Normal**

Student 16	Noise level: **4**	Noise level: **4**	Noise level: 7
	Luminosity level: **7**	Luminosity level: **2**	Luminosity level: 3
	State: **not understanding**	State: **not concentrating**	State: **not understanding**
	Stress: **stress**	Stress: **normal**	Stress: **stress**

Bold indicates the values of the different context parameters detected randomly by IoT devices.

**Table 3:** Example of local decision concerning student 5.

	Subject 1	Subject 2	Subject 3	Subject 4	Subject 5	Subject 6
Student 5	Turn on light	Decrease noise. You are absent.	Concentrate	Decrease noise	Decrease noise. Turn on light.	Relax

## Data Availability

No data were used to support this study.

## References

[1] Jih W.-R., Hsu J. (2009). Agent-based context-aware service in a smart space. *Agent-Based Ubiquitous Computing*.

[2] Ye D., Mei Y., Shang Y., Zhu J., Ouyang K. (2016). Mobile crowd-sensing context aware based fine-grained access control mode. *Multimedia Tools and Applications*.

[3] Chen R.-M. (2020). Whether economic freedom is significantly related to death of COVID-19. *Journal of Healthcare Engineering*.

[4] Pradhan B., Bhattacharyya S., Pal K. (2021). IoT-based applications in healthcare devices. *Journal of Healthcare Engineering*.

[5] Hameed K., Bajwa I. S., Sarwar N., Anwar W., Mushtaq Z., Rashid T. (2021). Integration of 5G and block-chain technologies in smart telemedicine using IoT. *Journal of Healthcare Engineering*.

[6] Alturki U. T., Aldraiweesh A., Kinshuck D. (2016). Evaluating the usability and accessibility of LMS “blackboard” at King Saud University. *Contemporary Issues In Education Research*.

[7] Beriswill J. (2018). *Zoom Redefines Web Conferencing for Education*.

[8] Jones N. (2006). E-college Wales, a case study of blended learning. *The Handbook of Blended Learning: Global Perspectives, Local Designs*.

[9] Truong H. M. (2016). Integrating learning styles and adaptive e-learning system: current developments, problems and opportunities. *Computers in Human Behavior*.

[10] Perales M., Pedraza L., Moreno-Ger P. Work-in-progress: improving online higher education with virtual and remote labs.

[11] Soonthornphisaj N., Rojsattarat E., Yim-Ngam S. (2006). Smart E-learning using recommender system. *Lecture Notes in Computer Science*.

[12] Sarwar S., Qayyum Z. U., García-Castro R., Safyan M., Munir R. F. (2019). Ontology based E-learning framework: a personalized, adaptive and context aware model. *Multimedia Tools and Applications*.

[13] Mayer R. E. (2017). Using multimedia for e‐learning. *Journal of Computer Assisted Learning*.

[14] Oxana K., Vladimir D., Pavlidis G. Upgrading the mobile distance learning system architecture.

[15] Sabagh A. A. A., Al-Yasiri A. (2015). GECAF: a framework for developing context-aware pervasive systems. *Computer Science - Research and Development*.

[16] Asabere N. Y. (2013). Towards a viewpoint of context-aware recommender systems (CARS) and services. *International Journal of Computer Science and Telecommunications*.

[17] Zaguia A., Tadj C., Ramdane-Cherif A. (2015). Context-based method using Bayesian network in multimodal fission system. *International Journal of Computational Intelligence Systems*.

[18] Tarus J. K., Niu Z., Mustafa G. (2018). Knowledge-based recommendation: a review of ontology-based recommender systems for e-learning. *Artificial Intelligence Review*.

[19] Udupi P. K., Malali P., Noronha H. Big data integration for transition from e-learning to smart learning framework.

[20] Priyahita R. The utilization of e-learning and artificial intelligence in the development of education system in Indonesia.

[21] Lone Z. A., Chawla P., Rana A. E-learning system architecture for cloud computing–a review.

[22] Ali S., Uppal M. A., Gulliver S. R. (2018). A conceptual framework highlighting e-learning implementation barriers. *Information Technology & People*.

[23] Gogo K. O., Nderu L., Mwangi R. W. Book fuzzy logic based context aware recommender for smart e-learning content delivery.

[24] Gleich D., Sarjaš A., Malajner M. Corela collaborative learning environment for electrical engineering education.

